The article "Neuroprotective Role of Intermittent Hypobaric Hypoxia in Unpredictable Chronic Mild Stress Induced Depression in Rats" was retracted in 2025. Reasons: duplicated images; overlap with earlier publications; original data or images not available; concerns about the images.

# Neuroprotective Role of Intermittent Hypobaric Hypoxia in Unpredictable Chronic Mild Stress Induced Depression in Rats

**DOI:** 10.1371/journal.pone.0149309

**Published:** 2016-02-22

**Authors:** Neetu Kushwah, Vishal Jain, Satayanarayan Deep, Dipti Prasad, Shashi Bala Singh, Nilofar Khan

**Affiliations:** Neurobiology Division, Defence Institute of Physiology & Allied Sciences, DRDO, Lucknow Road, Timarpur, Delhi-110054, India; CSIR-INSTITUTE OF GENOMICS AND INTEGRATIVE BIOLOGY, INDIA

## Abstract

Hypoxic exposure results in several pathophysiological conditions associated with nervous system, these include acute and chronic mountain sickness, loss of memory, and high altitude cerebral edema. Previous reports have also suggested the role of hypoxia in pathogenesis of depression and related psychological conditions. On the other hand, sub lethal intermittent hypoxic exposure induces protection against future lethal hypoxia and may have beneficial effect. Therefore, the present study was designed to explore the neuroprotective role of intermittent hypobaric hypoxia (IHH) in Unpredictable Chronic Mild Stress (UCMS) induced depression like behaviour in rats. The IHH refers to the periodic exposures to hypoxic conditions interrupted by the normoxic or lesser hypoxic conditions. The current study examines the effect of IHH against UCMS induced depression, using elevated plus maze (EPM), open field test (OFT), force swim test (FST), as behavioural paradigm and related histological and molecular approaches. The data indicated the UCMS induced depression like behaviour as evident from decreased exploration activity in OFT with increased anxiety levels in EPM, and increased immobility time in the FST; whereas on providing the IHH (5000m altitude, 4hrs/day for two weeks) these behavioural changes were ameliorated. The morphological and molecular studies also validated the neuroprotective effect of IHH against UCMS induced neuronal loss and decreased neurogenesis. Here, we also explored the role of Brain-Derived Neurotrophic Factor (BDNF) in anticipatory action of IHH against detrimental effect of UCMS as upon blocking of BDNF-TrkB signalling the beneficial effect of IHH was nullified. Taken together, the findings of our study demonstrate that the intermittent hypoxia has a therapeutic potential similar to an antidepressant in animal model of depression and could be developed as a preventive therapeutic option against this pathophysiological state.

## 1. Introduction

In humans, the development of different psychological conditions has been vividly influenced by the chronic exposure to stressful environment. Depression is one of the best examples of such condition. Depression is characterized by an inability to experience pleasure (anhedonia) and by general loss of interest and motivation. The onset of depression results from an interaction between the genetic predisposition and life stressors. Moreover, most episodes of major depression are preceded by stressful life events [1]. multiple stressful events substantially increase the risk of a depressive onset such as different psychological conditions. It is important to note that the chronic stress (ongoing for weeks or months) is a stronger predictor of depressive symptoms than the acute stressors [2]. Developing a perfect animal model to study depression is very complex as humans, unlike mice, lack observable traits of depression such as low self esteem, suicidal tendency etc.

Unpredictable chronic mild stress or UCMS has been widely used as a model of depression. This model has a high degree of predictive validity (behavioural changes are reversed with antidepressant drugs); face validity (chronic stress induces the behavioural alterations characterizing depressed patients), and construct validity (CMS decreases sensitivity in the brain reward system). Earlier studies show that many of the deteriorating effects of UCMS can be ameliorated by antidepressant agents [3–6]. In rodents, UCMS also has good face validity as it can elicit depression like symptoms such as lack of sucrose preference [6, 7] interpreted as anhedonia, a core symptom of depression [8]. Significant progress has been made in our ability to treat depression, but not all depressed patients respond to available antidepressants, and the therapeutic response requires several weeks or months of treatment [9, 10]. In addition, till date very limited information is available about the neurobiological alterations that underlie the pathophysiology or treatment of depression.

Intermittent hypoxia (IH) is an endogenous phenomenon in which sublethal hypoxic insult induces protection against future lethal hypoxia and other insults. IH can be beneficial to both human beings and animals. Both preconditioning and IH as reported earlier, exerts an endogenous protective mechanism that helps neurons survive further lethal insults. Although the mechanism involved in preconditioning and intermittent hypobaric hypoxia (IHH) are poorly understood [11]. Repeated episodes of hypobaric hypoxia interspersed with normoxic periods (IHH) have long been used for training pilots, mountaineers, and athletes, and even applied for treatment and prevention of human diseases such as hypertension, ischemic coronary artery diseases, Parkinson’s disease, and acute myeloid leukemia [12–15]. The hippocampus is one of the important brain areas which is associated with the cognitive functions like learning and memory, and is highly susceptible to stress and senescence [16, 17]. The acute and the chronic stress treatments have been reported to decrease brain derived neurotrophic factor (BDNF) mRNA levels throughout the hippocampus [10, 18, 19].

BDNF is the most prevalent neurotrophic factor in the brain, responsible, among the other functions, for neuronal survival, maintenance and growth. Levels of serum BDNF are known to be decreased in major depressive patients [19] and are associated with vulnerability to develop mood disorders in healthy subjects [20]. It has also been suggested that the reduced hippocampal cell numbers may be involved in the pathophysiology of depression [21] and treatment with antidepressants has been shown to increase hippocampal neurogenesis [22]. Neutrophic factors were initially characterized for regulating neuronal growth and differentiation during development, but were later found to be potent regulators of plasticity and survival of adult neurons and glia. Acute and chronic stress have been known to decrease the levels of BDNF in DG and hippocampus [23]. Antidepressant treatment increases the expression of BDNF in these regions [24], and can prevent the stress induced decrease in BDNF levels. Also, there is evidence that antidepressants enhance hippocampal BDNF levels in humans [25]. Several studies have examined the notion that BDNF–TrkB signalling has no effect on neurogenesis in adult brain. Even though few of those state that the manipulations of BDNF–TrkB signalling alter the differentiation of neuronal progenital cells NPCs [26], there are others who support the view that this signalling is important for the survival of NPCs [26, 27]. In the present study, we attempted to find out whether blocking the BDNF–TrkB signalling can reduce the expression of BDNF itself in hippocampus.

The possibility that BDNF is also involved in the pathophysiology of stress-related mood disorders is supported by reports that BDNF expression is decreased by exposure to stress [23, 28]. Hypoxic exposure may also result in neuronal cell death. Apoptosis is a normal physiological programmed cell death that can be enhanced or modulated by a variety of external stimuli, such as viral infections, medications, ischemia, hypoxic exposure and pathological condition, while necrosis, the other type of cell death is the result of severe injury to cell and the initiating events are more mechanical rather than biological unlike apoptosis. The neuronal death observed after ischemia/ hypoxia may be apoptotic or necrotic in nature and depends on nature of hypoxia. Severe and acute insult of hypoxia is related to necrotic cell death whereas the chronic exposure may cause the apoptotic death [29], which can be mediated via various pathways that cause condensation of the cytoplasm and chromatin, membrane blebbing, DNA fragmentation, and ultimate sequestration of cellular contents into membrane-bound apoptotic bodies but the necrotic signs are proliferation of ER, disaggregation of polyribosome and dendritic swelling [30, 31]. The present study is designed to explore the effect of IHH on depression like behaviour using unpredictable chronic mild stress induced depression as a model. Furthermore, the potential mechanisms underlying UCMS induced modulation of BDNF expression in hippocampus was also studied.

## 2. Material and Methods

### 2.1. Chemicals and Reagents

All the analytical chemicals were procured from sigma chemicals. Imipramine, Bovine serum albumin was purchased from Sigma Aldrich, (St Louis, USA). Rabbit polyclonal Primary antibodies for BDNF, DCX, NeuN, and Beta Actin were obtained from Abcam (Cambridge, USA). Anti rabbit Secondary antibodies were procured from Millipore (Darmstadt, Germany). Chemicals for western blot were procured from Bio-Rad (California, USA).

### 2.2. Ethics Statement

All experiments were conducted in accordance with the Committee for the Purpose of Control and Supervision of Experiments on Animals, Government of India. The experimental and animal 98 care protocol for this study was approved by Institutional Committee for Animal Care and Use (ICACU), of the Defence Institute of Physiology and Allied Sciences (27/1999/CPCSEA).

### 2.3. Animals

2–3 months old male sprague dawley rats (weight 180-200g) were used for the study. The animals were maintained in experimental animal facility under hygienic conditions with day and night cycle of 12 h each. Animals were divided into 8 groups (Table 1).All animal handling was performed between the time windows of 10.00 AM to 11.30 AM to avoid experimental deviations due to diurnal variations in corticosterone concentration. The temperature and humidity was maintained at 25±2°C and 65±5%, respectively. All surgical procedures were performed under kitamine/xylezine anesthesia and all efforts were made to minimize the pain or discomfort to the animals. Food and water available as *ad libitum*.

**Table 1:** Tabular representation of various treatments in different groups.

Group No	UCMS 24h/Day	IHH 4h/day	AD (IMIP) i. p. 10mg/kg/Day	K252a i. c. v. (50μg)
**1 (Control)**				
**2**		**+**		
**3**	**+**		**+**	
**4**	**+**			
**5**	**+**	**+**		
**6**	**+**		**+**	
**7**	**+**	**+**		**Vehc.**
**8**	**+**	**+**		**+**

### 2.4. Experimental Design

Experiment was performed in two phases in which Phase I include random division of rats in six different groups (n = 10/group). Out of six groups three groups kept in control conditions with Intermittent hypobaric hypoxia (IHH) or antidepressant treatment (Imipramine) and other three groups were exposed to Unpredictable Chronic Mild Stress (UCMS) with Intermittent hypobaric hypoxia (IHH) or antidepressant treatment (Imipramine) as shown in Table 1 and Fig 1. Rats were kept in standard cages (4 animals/cage) and acclimatized to experimental conditions for one week prior to experiments.

**Fig 1:** Schematic diagram to represents experimental design and time duration of different conditions (stress or interventions).

### 2.5. Unpredictable chronic mild stress (UCMS) protocol

UCMS was performed as suggested by Shalaby et al, with few modifications [32]. Briefly, seven unpredictable mild stresses were given sequentially for seven days (1 week) which consisted of a variety of mild stressors, including restraint, forced swim in ice-cold water (5 min), food and water deprivation (24 h), cage tilting (45°), reversal of the light/dark cycle, strobe light, and pairing with another stressed animal, in a fix schedule that lasted for 1 week and was repeated thereafter.

### 2.6. Intermittent Hypobaric Hypoxia protocol

Rats were given IHH as per protocol suggested by Zhu et al., with minor modifications [33]. Briefly, the animals were kept in a specially designed animal decompression chamber and were exposed to a simulated altitude of 5000 m (16,404 ft) by reducing the ambient barometric pressure, temperature was kept as 28±2°C and humidity kept at 60%. The total duration of experiment was two weeks with frequency of 4 hrs /day (during last 2 weeks of 5 weeks UCMS exposure).

### 2.7. Drug and inhibitor treatment

Imipramine, a well known antidepressant was used as positive control and was administered intraperitonealy (i.p.) at a dose of 10mg/kgbody weight /day, (dissolved in sterile 0.9% saline) for 14 days to both control as well as UCMS exposed group respectively. To determine the role of BDNF, we blocked BDNF-TrkB signalling using K252a. Intracerebroventricular (i.c.v) infusion of either vehicle (aCSF) or tyrosine K252a was done (50μM; dissolved in aCSF) into the right hemisphere via a cannula that was placed in the right lateral cerebral ventricle (1.0 anteroposterior relative to bregma, 1.5 mm lateral to the midline, and 3.4 mm deep to the pial surface). The cannula was cemented, and the incision was sutured. Four days after surgery, animals exposed to 2 weeks of IHH exposure.

### 2.8. Behaviour parameters

#### 2.8.1. Elevated Plus Maze (EPM)

The EPM is a rodent model of anxiety that is used as a screening test for putative anxiolytic compounds and as a general research tool in neurobiological anxiety research. The test settings consists of a plus shaped apparatus with two open and two enclosed arms, each with an open roof, elevated 40–70 cm from the floor. The model is based on the rodents’ aversion of open spaces. This aversion leads to the behaviour termed thigmotaxis, which involves avoidance of open areas by confining movements to enclosed spaces or to the edges of a bounded space. Rats were trained daily for 3–5 d before testing. Maze was cleaned and dried after each experiment. Individual transport cage containing rats was brought into the behavioural testing room; rodent was taken out of the cage and kept free at the junction of the open and closed arms, facing the open arm. Video-tracking system was started and time was set for 5 min when the rat was placed in the maze. The video-tracking system automatically recorded the number of entries made by the rodent into open and closed arms and the time spent in the open and closed arm were also monitored. Simultaneous manual recording of the number of arm entries and time spent in each open arm by the rats was done on the data sheets with timer.

#### 2.8.2. Open Field Test (OFT)

OFT was used to examine the anxiety and the locomotor activity of the rats for the 5 min reach trial. The apparatus consists of white plexiglass box 40x 40 cm with its floor divided in to 16 squares with squares as centre area and 12 squares as periphery. Rats were trained before starting the experiment and placed at the centre of the apparatus and activities were recorded with the video camera fixed above the apparatus.

#### 2.8.3. Force swim Test (FST)

FST was used to check the antidepressant activity of the rats. It is also called as behaviour despair test and is based on the observation that if rats develop an immobile posture in an inescapable cylinder filled with water. FST is a standardized test of depressive- like behaviour in which depression is inferred from increased duration of immobility, was conducted as described by O’ Connor [34]. The duration of immobility was determined during the test using the mobility function. Briefly, rats were plunged individually into a vertical plexi glass cylinder (40 cm high; 20 cm in diameter) filled with 30 cm deep water (20–25°C). After the 5 min period of the test, they were removed and allowed to dry. The duration of Immobility was measured for 5 min by an observer blind to the condition of the rats using the mobility function of ANY Maze software (Stoelting Co, USA). ANY Maze software was used for the acquisition and analysis of all the behaviour parameters.

### 2.9. Tissue processing

After completion of exposure and behaviour analysis rats were anesthetized with ketamine/xylazine, perfused transcardially with 1x Phosphate Buffer Saline (PBS), pH 7.4 and fixed in 4% paraformaldehyde (PFA) solution (dissolved in 1x PBS). Whole brain was isolated under aseptic conditions and was post fixed in same fixative PFA for 24 h then subjected to dehydration in 10%, 20%, and 30%, sucrose solution for 24 hrs. Sectioning was done in (30 μm thickness) cryostat (Leica 3050, Germany).

### 2.10. Embedding and sectioning

The processed brain samples were embedded in cryofluid and kept in the cryostat chamber at –25°C. Solidified gen was fixed on the cutting hood whose temperature being kept at -15°C then the 30 μm sections were cut from the hippocampus and collected in the 1x PBS with 0.02% sodium azide and placed in six well tissue culture plates.

### 2.11. Neuronal death analysis

#### 2.11a. Cresyl violet (CV) staining

After exposure, rats were anesthetized and perfused with ice cold PBS, fixed with 4% paraformaldehyde, cryoprotected in 30% sucrose solution, sliced into 10 μm free floating sections and processed for Cresyl violet staining. Morphology of neurons in CA1 regions was studied. Briefly every sixth section from each individual was taken, dehydrated using gradient alcohol concentration, stained with cresyl violet for 3 mins and then rehydrated again. The sections were transferred to slides and mounted with permanent mounting media. Morphology of neurons in CA1 region was observed under light microscopy. Counting of pyknotic/dead cells was done using freely available Image J software.

#### 2.11b. Neurodegeneration

Apoptosis is a marker for cellular self-destruction due to activation of nucleases that finally degrade the nuclear DNA into fragments of more or less 200 base pairs in length. Detection of these DNA fragments was done in tissue obtained after cryo- sectioning directly using TUNEL apoptosis detection kit (Millipore). TUNEL (Terminal deoxynucleotidyl Transferase Biotin-dUTP Nick End Labelling) identifies apoptotic cells *in situ*. Experiment was done as per the manufacturer’s instruction. Briefly, sections were washed with PBS for 30 min at 37°C. The sections were treated with proteinase K and incubated for 15–30 min at 37°C followed by washing with PBS four times for 2 min. Sections were then incubated with Tdt (Terminal deoxynucleotidyl Transferase) buffer for 5–10 min. Dark incubation of the sections with Tdt end labelling cocktails was done at 37°C for 60 min. Further sections were incubated with TB buffer (termination buffer) for 5 min at room temperature. All sections were washed with PBS for 2 min and blocking solution was added for 20 min. Avidin FITC solution was applied for 30 min at 37°C followed by washing with PBS for 15 min twice. Finally sections were mounted with antifade agent for long term storage and viewed under fluorescence microscopy (Olympus, Japan).

#### 2.11c. Neuronal density

neuronal density was assessed by expression of NeuN, a well established mature neuronal marker by IHC.

### 2.12. Immunohistochemistry (IHC)

Tissue sections were processed for IHC. The sections were washed twice with PBS prior to sodium citrate treatment at 100°C for 10 min for antigen retrieval, followed by washing with PBST 3x10 times (0.1% triton). All the sections were permeabilized in 0.25% PBST, washed with PBST 3x10 times (0.1% Triton X100). Rabbit polyclonal Primary antibody BDNF (1:500), doublecortin (1:500), NeuN (1:500) (Abcam, USA) was diluted in 5% normal goat serum (blocking solution) and added in each section and incubated for 48 h at 4°C, washed with PBST 3x10 times (0.1% triton). Anti rabbit secondary antibody (1:1000) was added for 2 h at room temperature, washed with PBST 3x10 times and sections were developed in the DAB. Alcohol treatment was done as 50%, 70%, 100%, followed by xylene treatment and sections were mounted in the DPX mounting medium and viewed under light microscopy.

### 2.13. Sample preparation for western blot analysis

Expression of BDNF at protein level in hippocampus was estimated by western blotting. Hippocampus samples for western blot were prepared as: 1 ml of lysis buffer with 2μl protease inhibitor cocktail and phosphatase inhibitor was added and homogenized in the sonicator at 4°C. Homogenate was centrifuged at 10000 g for 10 min at 4°C. Supernatant was collected for protein estimation and western blot experiments.

### 2.14. Immunoblotting

The protein content of the samples for western blot was estimated by Bradford [35] using BSA as the standard [36]. 60 μg of protein was resolved by electrophoresis in SDS-PAGE 10% polyacrylamide gels. Transferred to polyvinylidene fluoride membranes pre-soaked in transfer buffer using a semidry transblot module (BIORAD). The transfer of protein bands to the membrane was verified by Ponceau S Staining. The membrane was blocked and probed with 3% BSA blocking and Rabbit polyclonal BDNF 1:100 (Abcam, USA) respectively and incubated overnight at 4°C the membrane was washed with PBST (1x PBS, pH 7.4, 0.1% Tween 20) 3x 10 min and was incubated with HRP conjugated anti rabbit secondary antibodies for 2–3 h and developed in a x-ray through chemiluminiscence peroxidase Kit (Sigma, St. Louis, USA). The protein expression in each group was quantified by densitometry analysis.

### 2.15. Statistical Data analysis

All behavioural results were analysed by using AnyMaze software. 6–10 rats were taken for the behaviour study in each group. All behaviour parameters like time spent in targeted zone, number of entries and immobility duration was analyzed using AnyMaze software. Histological images were analysed using ImageJ software. TUNEL positive, Pycknotic and DCX positive cells were counted using cell counter option in ImageJ software. Mean pixel intensity was measured for BDNF and NeuN expression in desired region using Image J software. 6–7 individual observations were taken from each animal for the analysis.

All the data are expressed as mean ± SEM. Statistical analysis was performed using one-way ANOVA, with multiple intergroup comparisons made using Newman-Keuls post hoc test, throughout the study unless specified otherwise. The significance level for all tests was set at p < 0.05.

## 3. Results

### 3.1. IHH showed no neuronal damage unlike HH

The DNA fragmentation remains one of the characteristic markers for apoptosis. TUNEL staining preferentially labels apoptotic nuclei by binding of digoxigenin to the 3’ ends of the DNA breaks. To assess the effect of IHH on the neuronal health we measured the neuronal densities in CA1 region as well as the apoptotic injury through TUNEL assay. Results showed that IHH do not cause cell loss as no change in neuronal densities was found in hippocampus in group exposed to IHH as compared to control. In contrast; the exposure to HH significantly reduces the neuronal density as reported previously when compared to control group (Fig 2).

**Fig 2:** Effect of Hypobaric hypoxia (HH) and Intermittent Hypobaric Hypoxia (IHH). This figure represents Neuronal density (NeuN) and TUNEL positive cells in CA1 region of hippocampus during chronic Hypobaric hypoxia (HH) and Intermittent hypoxia (IHH) exposure. Data represents Mean + SEM. “*” represents p<0.05 when compared to control group.

Similarly, there was no significant differencefound in TUNEL positive cells in CA1 region of IHH group compared to control however the animals exposed to chronic HH showed abundant TUNEL positive cells (Fig 2).

### 3.2. IHH prevents UCMS induced depression like symptoms

After analyzing the effect of IHH under control conditions we further analyzed its efficacy against UCMS induced depression like symptoms. Five weeks of UCMS exposure led to increased anxiety and induces depression like symptoms when compared to control group as evident from increased immobility in FST, a widely used animal model for assessing antidepressant activity. There was no significant difference between control groups with and without IHH or drug treatment. The results showed that IHH treatment during UCMS exposure significantly reduced UCMS induced depressive behaviour as shown in FST analysis (Fig 3).

**Fig 3:** Immobility episodes in Force Swim Test (FST). This figure represents total immobility time in seconds in following groups (1) Control (2) Control + IHH (3) Control + Imipramine (4) UCMS exposed group (5) IHH treated during UCMS exposure and (6) Antidepressant (Imipramine) treated during UCMS exposed group. Data represents Mean + SEM. “***” and “**” represents p<0.001 and p<0.01 when compared to control and UCMS group respectively.

Similarly rats subjected to UCMS also consistently displayed increased anxiety-like behaviour on the elevated plus-maze (EPM). EPM analysis revealed that 5 week UCMS exposure significantly reduced number of entries and the total time spent in open arm (Fig 4) as compared to control, whereas providing IHH during last 2 weeks of UCMS exposure significantly ameliorated this abating effect of UCMS by increasing the total time spent and number of entries in open arms.

**Fig 4:** Anxious behaviour analysis in Elevated Plus Maze (EPM). This figure represents Number of entries and total time spent in open arms of EPM in following groups (1) Control (2) Control + IHH (3) Control + Imipramine (4) UCMS exposed group (5) IHH treated during UCMS exposure and (6) Antidepressant (Imipramine) treated during UCMS exposed group. Data represents Mean + SEM. “***” and “**” represents p<0.001 and p<0.01 when compared to control and UCMS group respectively.

Open Field Test (OFT) was used to assess the locomotory as well as the exploratory activity of rats. UCMS exposure shown to impede the exploring activity of rats as manifested by decreased number of entries and time spent (Fig 5) in central zone of OFT. On the other hand, the IHH treated group showed significant enhancement in the time spent and number of entries in central zone during OFT (Fig 5).

**Fig 5:** Locomotor and Exploratory activity analysis in Open Field Test (OFT). This figure represents Number of entries and total time spent in central zone of OFT in following groups (1) Control (2) Control + IHH (3) Control + Imipramine (4) UCMS exposed group (5) IHH treated during UCMS exposure and (6) Antidepressant (Imipramine) treated during UCMS exposed group. Data represents Mean + SEM. “***” and “**” represents p<0.001 and p<0.01 when compared to control and UCMS group respectively.

### 3.3. IHH provides protection against UCMS induced neuronal loss

NeuN is a well know neuronal marker used to identify mature neurons. In present study it was found that the UCMS reduces the neuronal density in CA1 region of hippocampus (Fig 6) where as the IHH treatment during last 2 weeks of UCMS exposure significantly ameliorated this neuronal loss. Neuronal density in IHH group was found comparable to the Imipramine treated group which was taken as positive control for antidepressant. Correlated observations were seen in the drug treated and IHH treated group. While, there was no significant change observed in IHH treated group during control condition and control group.

**Fig 6:** Effect of IHH treatment on Neuronal density. This figure represents densitometric analysis of NeuN, well known mature neuronal marker in following groups: (1) Control (2) Control + IHH (3) Control + Imipramine (4) UCMS exposed group (5) IHH treated during UCMS exposure and (6) Antidepressant (Imipramine) treated during UCMS exposed group. Data represents Mean + SEM. “***” and “**” represents p<0.001 and p<0.01 when compared to control and UCMS group respectively.

Furthermore, the neuronal cell loss was assessed using CV staining and it was observed that in group exposed to UCMS there was a significant increase in the number of pyknotic cells in CA1 region of the hippocampus when compared to control groups (Fig 7). Whereas IHH treatment after UCMS exposure reduced the number of pyknotic cells significantly when compared to UCMS exposed group alone (Fig 7). No significant difference was found in IHH and drug treated groups.

**Fig 7:** Effect of IHH treatment Neuronal cell morphology through CV staining. This figure represents change in number of pycknotic cells in CA1 region of hippocampus through Cresyl violet (CV) staining in following groups: (1) Control (2) Control + IHH (3) Control + Imipramine (4) UCMS exposed group (5) IHH treated during UCMS exposure and (6) Antidepressant (Imipramine) treated during UCMS exposed group. Data represents Mean + SEM. “***” and “**” represents p<0.001 and p<0.01 when compared to control and UCMS group respectively.

Similarly, UCMS exposure for 5 weeks was found to substantially increase DNA fragmentation in the CA1 region as revealed by increased number of TUNEL positive cells. Administration of IHH during last 14 days of UCMS exposure on the other hand significantly decreased the number of TUNEL positive cells when compared to group exposed to UCMS alone (Fig 8). No significant changes were observed in groups treated with IHH or Imipramine in control conditions.

**Fig 8:** Effect of IHH treatment on Apoptosis through TUNEL staining. This figure represents change in number of TUNEL positive cells in CA1 region of hippocampus through TUNEL staining in following groups: (1) Control (2) Control + IHH (3) Control + Imipramine (4) UCMS exposed group (5) IHH treated during UCMS exposure and (6) Antidepressant (Imipramine) treated during UCMS exposed group. Data represents Mean + SEM. “***” and “*” represents p<0.001 and p<0.05 when compared to control and UCMS group respectively.

### 3.4. IHH enhances the adult neurogenesis in hippocampus

To determine whether adult neurogenesis contributes to this neuroprotective effect of IHH, we studied DCX expression in hippocampus. It was observed that there was decrease in the number of DCX+ cells in DG region of hippocampus in comparison to control group. On the contrary, the IHH treatment reverted back this effect by substantially increasing the number of DCX+ cells in hippocampus and were comparable to Imipramine treated group. Also, there was no significant changes found between control and IHH treated group in control conditions (Fig 9).

**Fig 9:** Effect of IHH treatment on adult neurogenesis. This figure represents change in number of Doublocortin (DCX) positive cells in DG region of hippocampus in following groups: (1) Control (2) Control + IHH (3) Control + Imipramine (4) UCMS exposed group (5) IHH treated during UCMS exposure and (6) Antidepressant (Imipramine) treated during UCMS exposed group. Data represents Mean + SEM. “***” represents p<0.001 when compared to control and “**”, “#” represents p<0.01 and p<0.05 when compared to UCMS group.

### 3.5. Role of BDNF in IHH mediated neuroprotection

BDNF is directly involved in neurite outgrowth and regulates the survival, growth, differentiation, and maintenance of neurons. BDNF is the essential neurotrophic factor that has been implicated in adult neurogenesis as well. It is also known to play role in neuroprotection and in neurogenesis related pathways. In present study we hypothesized that BDNF may play important role in IHH mediated neuroprotection. BDNF expression analysis through immunoblotting revealed the reduced BDNF level in UCMS exposed groups than control group, though the level got conversely increased when IHH was provided during last 14 days of UCMS exposure (Fig 10) Similar pattern was observed in differential expression analysis of BDNF in CA1 region of hippocampus through Immunohistochemistry (Fig 10) However, no significant changes were found in the Imipramine treated group and control group.

**Fig 10:** Effect of IHH treatment on BDNF immunoreactivity in hippocampus. This figure represents change in BDNF expression in whole hippocampus through immunoblotting (A) as well as in CA1 region through immunohistochemiustry (B) in following groups: (1) Control (2) Control + IHH (3) Control + Imipramine (4) UCMS exposed group (5) IHH treated during UCMS exposure and (6) Antidepressant (Imipramine) treated during UCMS exposed group. Data represents Mean + SEM. “***” and “**” represents p<0.001 and p<0.01 when compared to control and UCMS group respectively.

Further to explore the role of BDNF in IHH mediated neuroprotection we blocked the BDNF signalling by K252a, a potent TrkB receptor (BDNF receptor) inhibitor. Blocking the TrkB signalling during IHH treatment in UCMS exposure showed remarkable findings. We observed that the blocking of TrkB receptor function nullifies the protective effect of IHH during UCMS exposure as evident from decreased time spent and number of entries in central zone of OFT (Fig 11A) as well as open arm of EPM (Fig 11B) and increasing immobility in FST (Fig 11C) when compared to group with IHH treatment during UCMS exposure alone. Similarly, the neuronal loss was also increased after blocking TrkB signalling during IHH treatment as number of TUNEL positive and pyknotic cell was dramatically increased in CA1 region of hippocampus in comparison to vehicle treated group. Also NeuN expression followed the same pattern as evident from decreased density of neurons in CA1 region of hippocampus on TrkB inhibition (Fig 12).

**Fig 11:** Effect of TrkB inhibition during IHH treatment on behavioural parameters. This figure represents effect of TrkB inhibition with K252a, a potent inhibitor of TrkB receptor, on IHH induced beneficial effect against UCMS exposure. Different behaviour parameters i.e. OFT (A), EPM (B) and FST (C) was studied after TrkB inhibition in following groups (1) IHH treated during UCMS exposure with vehicle and (2) IHH treated during UCMS exposure with K252a treatment (250mM). Data represents Mean + SEM. “***” represents p<0.001 when compared to vehicle group.

**Fig 12:** Effect of TrkB inhibition during IHH treatment on morphological parameters. This figure represents effect of TrkB inhibition with K252a, a potent inhibitor of TrkB receptor, on IHH treated group. Following TrkB inhibition both (vehc and K252a treated) groups were analyzed for (i) TUNEL +ve cells (ii) Pycknotic cells thorugh CV staining (iii) Neuronal density via NeuN immnoreactivity (iv) BDNF expression and (v) DCX +ve cells, in CA1 region of hippocampus. Data represents Mean + SEM. “***” represents p<0.001 when compared to vehicle group.

TrkB inhibition during IHH treatment also nullifies the IHH mediated enhancement of adult neurogenesis by significantly decreasing the number of DCX positive cells in DG region of hippocampus (Fig 12) Interestingly, our finding also showed that inhibition of BDNF mediated TrkB signalling, in reverse, reduces the expression of BDNF itself in hippocampus, even in the presence of IHH during UCMS exposure (Fig 12). This finding highlights the loop mechanism in BDNF synthesis in cell in response to stress or treatment.

## 4. Discussion

The primary findings of the present study are that UCMS, a well known model of depression causes congnitive decline and depression like symptoms whereas IHH showed ameliorating potential against detrimental effect of UCMS. In addition to providing neuroprotection, IHH was also found to enhance the neurogenesis in hippocampus against UCMS. Finally, the involvement of BDNF is explored in neurogenic and antidepressant like effect of IHH.

Depression is a condition of low mood and aversion to activity that can affect a person's thoughts, behaviour, feelings and sense of well-being. Major depression and anxiety disorders are associated with functional and morphological alterations in brain, along with symptoms reflecting both cognitive dysfunction and anxiety [37]. Clinical studies have shown that stressful life experiences are important etiological factors in the development and maintenance of depression and affective disorders [38, 39], particularly associated with cognitive and emotional biases [40, 41]. Severe hypoxic conditions are known to have lethal effects; on the other hand milder levels of oxygen desaturation may have beneficial effects [42]. The actual protocol to achieve intermittent hypoxia used in different studies varies greatly in cycle length, the number of hypoxic episodes per day and days of exposure, as well as being with or without hypobaric. Persuasive outcomes of intermittent hypoxia therefore may be linked to type of an exact protocol used in particular study. Keeping these points in mind we developed a protocol to use hypobaric hypoxia at an altitude of 5000m in intermittent episodes as intervention against UCMS induced depression like symptoms.

UCMS has long been used as a model of depression and their pathophysiological machinery such as decreased neurogenesis and HPA axis alterations [43]. Exposure to chronic stress can affect the development of certain forms of depression in humans and animal models [44, 45]. In present study UCMS is used as stress model to induce depression where we found that UCMS exposure for 5 weeks causes cognitive decline and depression like symptoms in EPM, FST and OFT. UCMS decreases number of entries and time spent in central zone of OFT and open arm of EPM with concomitant enhanced immobility episodes in FST. These results are in agreement with several other studies which showed that UCMS causes cognitive decline and depression like behaviour in animal models [45, 46]. On the other hand our findings showed that IHH ameliorate this depression like behaviour of animals by reducing immobility episodes in FST, and increasing exploratory activity in OFT. Similarly, IHH significantly enhanced the activity in open arms EPM. Our results, along with the previous reports, thus clearly indicated that IHH prevents the depressive anxiety like behaviour in various behavioural tests [42, 47].

Chronic hypobaric hypoxia leads to neurodegeneration in rat brain [48], altered neurotransmitter synthesis, uptake and release and changes in gene expression and protein functions. Out of different regions hippocampus is more prone to HH stress and in hippocampus CA1 region is highly vulnerable. Similarly UCMS known to impaired memory performance and inhibited autophagic flux causing apoptosis in CA1 region of hippocampus [49]. On the contrary IHH works through several defence mechanisms. There were various defensive properties of IHH on the improvement of depressive states in rat models [47]. IHH enhances the cell survival and neuronal differentiation [50]. Mild episodes of brief hypoxia show protective action against neuronal damage induced by hypoxia. Reports have shown the neuroprotective effects of IHH in nissle staining and TUNEL staining in hippocampal neurons [51]. In concomitant to these findings our study also showed that IHH prevents UCMS induced apoptosis by decreasing the number of pycknotic and TUNEL positive cells in hippocampal CA1 region which was however increased in UCMS treated groups. This is consistent with previous results by others showing that IHH can suppress apoptosis in the hippocampus and temporal cortex [51, 52]. The precise mechanisms by which IHH prevent apoptosis are, however, not well known. Indeed, it has been shown that IHH can exert neurotophic or neuroprotective effects via cell survival and growth factors such as BDNF, anti apoptotic protein; Bcl2, preserving mitochondrial membrane potential, increasing brain antioxidant capacity and Hypoxia-Inducible Factor and Erythropoietin [53–56]. Additionally IHH maintains neuronal density in hippocampus as apparent from improved NeuN density in CA1 region of hippocampus in comparison to UCMS exposed rats.

In many neurological disorders like Alzheimer’s or Parkinson’s and injury such as stroke [57–59] result in permanent loss of neurons with no prospect of cellular regeneration [60]. Neurogenesis is the progression of generating new neurons from neural stem cells and progenitor cells [61]. The DG is majorly having ability to produce new neurons in adulthood. Reduce neurogenesis in animal models have already been reported in depression studies [62]. Studies have shown that IHH increases the neurogenesis in DG region of the hippocampus [33]. We observed the similar findings as IHH increases the expression of DCX and NeuN positive cells in DG region of hippocampus whereas it decreased in UCMS treated rats so it can be postulated that increase neurogenesis may account for protective mechanism of IHH to cope up UCMS induced neuronal loss.

BDNF one of the most prevalent neurotrophic factors in the adult brain. Acute and chronic stress decrease levels of BDNF in different region of hippocampus [23]. A decreased expression of BDNF appears to be associated with depression like symptoms in animals and with depression symptoms in humans. A decreased serum BDNF level has been reported in human depression [63] and has been found to be an indicator of vulnerability to develop depression [64]. Several other animal models of depression have shown a reduced expression of BDNF in different brain regions (e.g. footshocks, cold swim, restraint stress, social defeat, learned helplessness, Chronic mild stress [23, 65–68]. In the present study, the expression of BDNF protein showed a significant decrease after UCMS exposure. Decreased BDNF levels have been previously reported, after acute and chronic mild repeated stress, chronic mild stress in hippocampus [69]. The results of the present study demonstrate that IHH induced an increase in the expression of BDNF in the hippocampus are in agreement with study by Zhu et al which showed that IH showed antidepressant like effect and enhance neurogenesis through BDNF mediated signalling [33]. Moreover, biological and pharmacological inhibitions of BDNF–TrkB signalling blocked the neuroprotective, neurogenic and antidepressant like effects of IHH, suggesting IHH neuroprotective nature may involve BDNF-TrkB signalling. Several studies have examined the effects that BDNF–TrkB signalling has no effect on neurogenesis in adult brain. Even though few states that manipulations of BDNF–TrkB signalling alter the differentiation of neuronal progenitor cells NPCs [26], many do show that this signalling is important for the survival of NPCs [26, 27]. The discrepancy between these reports and our findings can be explained by the fact that IHH may induce several other unknown factors which may lead to the added effects that what we observed in our study.

In addition to all these findings we also observed that blocking BDNF–TrkB signalling also reduces the expression of BDNF itself in hippocampus. This findings may attribute to loop mechanism in BDNF synthesis which explains how BDNF up-regulated its own transcription and translation as supported by several other studies which shows that BDNF stimulates its own transcription through promoter IV in cortical cell culture as well as in visual cortex [70, 71].

In summary, the present study demonstrates that IHH prevents UCMS induced depression like behaviour by enhancing hippocampus neurogenesis and BDNF–TrkB signaling in adult rats. These findings offer the challenging suggestion that deeply understanding the molecular and cellular mechanisms underlying physiological responses to IHH could provide novel targets for the safer and better treatment of neurological disorders which involves depression like symptoms.
